RETRACTED

# FNDC1 Promotes the Invasiveness of Gastric Cancer *via* Wnt/β-Catenin Signaling Pathway and Correlates With Peritoneal Metastasis and Prognosis

**DOI:** 10.3389/fonc.2020.590492

**Published:** 2020-12-17

**Authors:** Tao Jiang, Wenyu Gao, Shengjie Lin, Hao Chen, Bin Du, Qing Liu, Xiaoyan Lin, Qiang Chen

**Affiliations:** ^1^ Department of Medical Oncology, Fujian Medical University Union Hospital, Fuzhou, China; ^2^ Department of Digestive, Fujian Medical University Union Hospital, Fuzhou, China

**Keywords:** gastric cancer, FNDC1, peritoneal metastasis, prognosis, Wnt/β-catenin signaling pathway

## Abstract

**Background:**

Gastric cancer (GC) has a high morbidity and mortality rate, with peritoneal metastasis (PM) identified as the main site of metastasis. Our previous study found that FNDC1 has a higher frequency of mutations in patients with PM by high-throughput sequencing assay, suggesting that it may be associated with GC invasion and PM, however the specific mechanism remains unclear.

**Methods:**

First, the correlation between FNDC1 and PM and prognosis of GC was clarified by bioinformatics and clinicopathological analysis. Next, the effect of FNDC1 expression on the invasion and metastasis ability of GC was investigated *in vivo* and *in vitro*. Finally, the signaling pathways involved in the regulation of FNDC1 were explored.

**Results:**

FNDC1 was highly expressed in GC and was associated with PM and poor prognosis. FNDC1 was also associated with epithelial-mesenchymal transition (EMT) in GC cells. Through *in vivo* and *in vitro* experiments, it was clarified that knockdown of FNDC1 could inhibit the proliferation, invasion, and migration of GC cells. In addition, it was elucidated that FNDC1 promotes EMT through the Wnt/β-catenin signaling pathway.

**Conclusion:**

FNDC1 may be associated with the invasion of GC and PM after surgery. FNDC1 was highly expressed in GC tissues and cell lines, while significantly associated with poor DFS and OS in GC patients. Both univariate and multivariate analyses suggested that the expression of FNDC1 was an independent factor for GC. Knockdown of FNDC1 also significantly inhibited the proliferation, migration, and activity of GC cells. FNDC1 may promote EMT in GC cells through the regulation of Wnt/β-catenin signaling pathway. FNDC1 has the potential to be used as a predictor of PM and may also be studied in depth as a therapeutic target for GC, which has potential clinical utility and is worthy of further validation.

## Background

Gastric cancer (GC) is a common malignant tumor of the digestive tract, ranking fifth in tumor incidence and third in mortality worldwide (1). Although the prognosis of patients with GC is currently improved by radical surgery combined with postoperative adjuvant therapy, about 50% of patients experience tumor recurrence and metastasis within 2 years after surgery, eventually dying (2). Peritoneal metastasis (PM) is the most common site of metastasis in GC cases, and the "seed-soil" theory reasonably elaborates the process of PM formation (3). In this process, the invasion and metastasis of GC cell (seed) plays an important role. At present, there remains a lack of effective predictors of PM, and the prognosis of patients is very poor due to the limited treatment and efficacy. Therefore, the risk factors for PM require a more comprehensive analysis. In our previous study (4), the molecular characteristics and metastasis markers of Chinese GC patients were analyzed. Specifically, tumor and adjacent normal tissue samples were collected from GC patients after radical resection for whole exome sequencing (WES). The sequencing results were compared with the occurrence of PM and multiple genes potentially related to PM were selected, of which fibronectin type III domain containing 1 (FNDC1, also known as AGS8) had a higher frequency of mutations in PM patients. The results suggested that FNDC1 may be related to GC invasion and PM, however, its specific mechanism of action is still unclear.

RETRACTED

The FNDC1 gene, located on human chromosome 6q25.3, is a class of receptor-independent activators of G protein signal transduction that can activate G protein signaling through interactions with Gβγ subunits. Its encoded products can be involved in the construction of protein multimers and are expressed in different tissues such as the thyroid gland, heart, kidney, and the digestive tract. Several studies have found that FNDC1 is closely related to the development of many diseases including various tumors (5–7). Recent studies have reported a correlation between the expression of FNDC1 in GC and clinical characteristics of patients (8–10). However, the exact role of FNDC1 in GC and the potential molecular mechanism has not been fully elucidated, and the effect of FNDC1 on PM remains to be revealed.

On this basis, this study focused on the effect of FNDC1 expression on the invasive ability and PM of GC. We applied biological information analysis, gene transfection, RNA interference, proteomics, and tumor xenograft models to deeply analyze the function and mechanism of FNDC1 in the malignant biological behavior of GC.

## Materials and Methods

### Bioinformatic Analysis

Bioinformatic analysis was performed using R (version 3.6.1) and the associated Bioconductor package. GSE62254 expression profiling data were acquired from the GEO (https://www.ncbi.nlm.nih.gov/geo/query/acc.cgi?acc=GSE62254) (11). The Cancer Genome Atlas (TCGA) expression profile data were obtained through University of California, Santa Cruz (UCSC) Xena (https://xena.ucsc.edu/) (12). GSE62254 data were normalized using the Affy R package (13), and TCGA data were processed using the edge R package for normalization (11, 14, 15). Differentially expressed genes (DEGs) were identified using the limma R package with correction P < 0.05 and |logFC| > 1 (13, 16). Gene expression profiles were enriched by GSEA with adjustment for multiple testing using the Benjamini-Hochberg procedure (17).

RETRACTED

### Clinical Specimens

Formalin-fixed tumor tissues and paired adjacent normal tissues (5 cm from tumor edges) from 74 patients (54 males, 20 females; age range 25–71 years) were used for immunohistochemical analysis. All patients received radical surgery for primary GC at the Department of Gastric Surgery, Fujian Medical University Union Hospital from 2015 to 2016. The project was reviewed and approved by the Fujian Medical University Union Hospital Ethics Committee. Informed consent was obtained from all participants included in the study.

### Cell Culture, Plasmid Construction, and Infection

Five gastric cell lines (GES1, AGS, HGC27, BGC823, and MGC803) were purchased from the American Tissue Culture Collection (ATCC, Rockville, MD, USA). GES1, HGC27, BGC823, and MGC803 and were cultured in Dulbecco’s modified Eagle’s medium (Gibco, NE, USA), and AGS were cultured in F-12 Medium (Gibco, NE, USA). All cell lines were supplemented with 10% fetal bovine serum (Gibco) and 100 U/L penicillin-streptomycin solution at 37°C in a humidified atmosphere containing 5% CO2. Lentivirus, pGV493-hU6-MCS-CBh-gcGFP-IRES-Puro, pCDH-CMV-FNDC1-EF1-Puro, and pCDH-CMV-β-catenin-EF1-Puro were purchased from BIORN (Nanjing, China). The shRNA-FNDC1 sequence was 5-CCGAAGGGAAGGCGTAGATAA-3, and the lentivirus without the transgene was used as a negative control (NC). For viral particle generation, cloned DNAs and lentiviral packaging Mix (Jikai, Nanjing, China) were transfected into 293T cells using transfection reagent (GeneChem, Shanghai, China) in Opti-MEM media (Gibco; Thermo Fisher Scientific, Inc.). Transfection was performed in HiTransG medium when cells density reached 70–80%, according to the manufacturer’s protocols. After the lentivirus vector was transfected into the AGS, MGC803, and BGC823 cells, stable cell lines were obtained with puromycin treatment. Then the cells were divided into the following groups according to different treatment conditions, AGS control group: AGS cells without treatment; AGS-shRNA-NC group: transfected with GV493-shRNA-NC; AGS-shRNA-FNDC1 group: transfected with GV493-shRNA-FNDC1; MGC803 control group: MGC803 cells without treatment; MGC803-shRNA-NC group: transfected with GV493-shRNA-NC; MGC803-shRNA-FNDC1 group: transfected with GV493-shRNA-FNDC1; MGC803-shFNDC1 + β-catenin NC group : transfected with pCDH-CMV-EF1-Puro; MGC803-shFNDC1 + β-catenin group : transfected with pCDH-CMV-β-catenin-EF1-Puro; BGC823 control group: BGC823 cells without treatment; BGC823-FNDC1-NC group: transfected with pCDH-CMV-EF1-Puro; BGC823-FNDC1 group: transfected with pCDH-CMV-FNDC1-EF1-Puro; GES1 control group: GSE1 cells without treatment.

RETRACTED

### Immunohistochemistry

Tissues were fixed in formalin, embedded in paraffin, and sectioned before being mounted on slides which were then subjected to de-paraffinizing and rehydrating. Tissue antigen retrieval was performed using EDTA high-temperature water boiling at pH 9.0. Endogenous peroxidase activity was blocked by adding 50 μl of 3% hydrogen peroxide to each section. Fifty μl of non-immune goat serum was added to each section, followed by 50 μl of FNDC1 antibody (Bioss, Beijing, China) for 60 min at room temperature. Sections were rinsed three times with PBS and 50 μl of MaxVisionTM (KIT-5005 MaxVisionTM HRP-Polymer anti-rabbit IHC Kit) reagent was added. An appropriate amount of diaminobenzidine (DAB) color solution was added to the slide to cover the tissue completely. The intensity of staining was divided into four scales: 0 (negative, −), 1 (weak, +), 2 (moderate, ++), and 3 (strong, +++). In addition, the proportion of staining was graded as follows: 0 (<5%); 1 (5–25%); 2 (26–50%); 3 (51–75%); and 4 (>75%). The staining score was calculated by multiplying staining intensity with cell percentage. A staining score below 5 indicated low FNDC1 expression while a score above 5 was considered high FNDC1 expression.

### Quantitative Real-Time Polymerase Chain Reaction

Total RNA was extracted from cells with Trizol (Takara, Japan) and reverse transcribed with IScript cDNA synthesis kit (Bio-Rad, Hercules, CA, USA) according to the manufacturer's protocol. The PCR primer sequences were as follow: FNDC1-forward: 5’-CAACATTGCCTATG

GGAAGTCA-3’, FNDC1-reverse: 5’-CTCGATCCATTCACCTCCAG-3’; β-catenin-forward: 5’-GAAGGTCTGAGGAGCAGCTT-3’, β-catenin-reverse :5’-GCCATTGTCCACGCTGGATT

-3’; GAPDH-forward: 5’-CCCAACGATGCGGATATGGA-3’, GAPDH -reverse: 5’-TTCCCGTT

CTCAGCCTTGAC -3’. β-actin-forward: 5’-CTTCGCGGGCGACGAT-3’, β-actin- reverse : 5’- CCACATAGGAATCCTTCTGACC -3’. GAPDH and β-actin was regarded as an internal control. PCR was performed with SsoFast EvaGreen SuperMix (Bio-Rad, Hercules, CA, USA) and the fluorescence was measured using the Light Cycler 480 RT-PCR System (Roche Applied Science) by following the manufacturer’s instructions. The relative amount of each cDNA was determined by 2−ΔΔCt method and at least three independent biological replicates were included for each reaction.

RETRACTED

### Western Blot

Total proteins were extracted from cells infected or uninfected by lentivirus, and their concentrations were measured by BCA protein assay kit (Beyotime Biotechnology, Shanghai, China). Next, cell lysates were loaded on SDS-PAGE for separation and transferred onto the PVDF membrane (Millipore, Schwalbach, Germany). After incubation with relevant primary antibodies at 4°C overnight, the membrane was incubated with species-matched secondary antibodies. The antibodies used included the following: Anti-FNDC1 (1:2,000, HPA030963, Lot:#027M4006V, Sigma), Anti-GAPDH (1:5,000, ab181602, Lot:#GR43631-4, Abcam), Anti-E-cadherin antibody (1:1,000 CST, Boston, USA), Anti-vimentin antibody (1:1,000 CST, Boston, USA), Anti-Krt12 antibody (1:5,000 Abcam, Cambridge, UK), Anti-survivin antibody (1:5,000 Abcam, Cambridge, UK), Anti-Snail antibody (1:500 Abcam, Cambridge, UK), Anti-Slug antibody (1:500 Abcam, Cambridge, UK), and Anti-β-catenin antibody (1:10,000 Abcam, Cambridge, UK). The immune-reactive protein bands were visualized by ECL kit (Thermo Fisher Scientific, Pittsburgh, PA, USA).

### Cell Proliferation and Colony Formation

The cells in logarithmic growth phase were collected, seeded in 96-well plates at 4,000/well and cultured. After 12 h, the cell attachment time was set as 0 h. Five parallel samples were made at each time point, and 10 μl of Cell Counting Kit-8 (CCK-8, Beyotime Biotechnology, Shanghai, China) solution was added to each well at the specified times: at 0, 24, 48, and 72 h, respectively. The absorbance at 450 nm was measured with a microplate reader, and the absorbance obtained at each time was compared with the absorbance value at 0 h to draw a cell proliferation curve. For colony formation assay, 500 cells/well were inoculated into six-well plates and cultured for 7 days. An addition of 5 ml of 4% paraformaldehyde was made to fix the cells for 15 min, after which the fixative was discarded and the appropriate amount of GIMSA was added for staining for 30min. The GIMSA staining solution was then slowly washed off with running water and fixed cells were dried in an oven. The number of clones with greater than 10 cells was counted with a microscope.

### Cell Cycle Detection by Flow Cytometry

Cell cycle detection kit (BD biosciences, NY, USA) was used for detection. The transferred cells were collected after 48 h and centrifuged at 1,000 r/min for 5 min at 4°C. Cells were resuspended in 125 μl trypsin buffer and the reaction was carried out at room temperature for 10 min. Subsequently, 100 μl trypsin inhibitor and RNase buffer solution were added and incubated at room temperature for 10 min. Finally, 100 μl PI solution was added and incubated on ice in the dark for 10 min. Cell cycle distribution was analyzed by flow cytometry within 1 h of the final reaction.

RETRACTED

### Cell Migration and Invasion Assay

Cell migration and invasion ability were analyzed using a 24-well transwell chamber with 8 um polycarbonate membranes (Millipore, Washington, DC, USA). For the cell invasion assay, the chamber above the membrane was coated with Matrigel (40 μl/well) (Sigma-Aldrich) and then air-dried for 2–4 h at 37°C. Serum-free medium was used to adjust the cell density to 2.5 × 10^5^ cells/ml, and 100 μl of individual cells was added to the upper chamber along the wall, and the lower chamber was filled with 12% FBS (AGS: F12K medium, MGC803 and GES1: DMEM medium). After incubating for 24 h, cells that passed through the membranes were fixed with paraformaldehyde and dyed with Crystal Violet (Aladdin Biochemistry, Shanghai, China). The cells on the surface of the upper chamber were removed with a cotton swab. The cells in the lower chambers were counted in five random fields. Each condition was repeated in triplicate.

### EDU Cell Proliferation Assay

Cells in the logarithmic growth phase before or after transfection were seeded at 4 × 10^4^ cells per well in 96-well plates and cultured for 24 h. An addition of 100 μl of diluted Edu medium (1,000:1, Ribo Life Science, Suzhou, China) was made to each well and incubated for 2 h. After adding 50 μl of 2 mg/ml glycine, 100 μl of 1 × Apollo staining reaction solution was added to each well, protected from light, and incubated at room temperature on a de-staining shaker for 30 min. An additional 100 μl of penetrant was used to decolorize and wash three times, 10 min each time. An appropriate amount of 1 × Hoechst 33342 reaction solution was prepared, and 100 μl was added to each well and incubated on a shaker at room temperature for 30 min in the dark. Each well was washed three times with 100 μl PBS and immediately examined by confocal laser scanning microscopy (LSM800 confocal laser scanning microscope, Carl Zeiss AG, Germany).

### Co-Immunoprecipitation Assay

RIPA lysis buffer was added to the cells and centrifuged at 14,000 g for 15 min. Protein A/G-agarose spheres were prepared into 50% protein A/G-agarose working solution with PBS. A ratio of 100 μl was added to the sample per 1 ml, and 50% Protein A/G agarose working solution was added and centrifuged at 14,000 g for 15 min at 4°C. The concentration of total protein was determined using the BCA method, and the total protein was diluted to 3 μg/μl with PBS. Then, 5 μl of antibody (β-catenin 1:50) was added (IgG antibody was added to the control group) to make a final volume of 500 μl and 100 μl of protein A/G-agarose microspheres were added to capture the antigen-antibody complex, centrifuged at 14,000 g for 5 s, after which the protein A/G-agarose microsphere-antigen-antibody complex was collected. The sample was resuspended in an appropriate volume of loading buffer and the sample was boiled for 5 min to denature the pellet. The sample was detected by WB method using the antibody (β-catenin 1:5,000, ubiquitin 1:2,000).

RETRACTED

### Xenograft Tumor Formation Study

All animal work involving Xenograft Tumor Formation was approved by the Fujian Medical University Animal Care & Use Committee, Fujian, China. A total of 18 BALB/c (nu/nu) mice (body weight 16–18 g, male) were obtained from the Animal Model Center of Nanjing University and housed in a SPF grade environment [animal certificate number: SCXK (Su) 2015-0001]. Adaptive feeding was allowed for 7 days before inoculation. Cells were retrieved in logarithmic growth phase, prepared at a concentration of 5 × 10^7^ cell/ml and inoculated at 0.2 ml/mouse in the right armpit to establish a xenograft model. The diameter of the transplanted tumor was measured with a vernier caliper and randomized after the tumor size reached 100 mm^3^. Tumor diameter and mouse body weight were measured every 3 days. After 6 weeks, all mice were sacrificed by carbon dioxide method. Tumors were enucleated, weighed, and measured by volume. The calculation formula for tumor volume (TV) = 1/2 × a × b^2^, where a and b indicate the length and width, respectively.

### Statistical Analysis

Bioinformatic analysis was performed using the R package and Cytoscape. A survival curve was plotted by the Kaplan-Meier method and a log-rank test was used to compare the survival curves. Chi-squared tests or Fisher’s exact test was applied to the quantitative data, the t-test was used to compare mean values between the two groups, and one-way analysis of variance was used to compare the mean values between multiple groups. Univariate and multivariate analysis were plotted by a Cox proportional hazards model. All statistical analyses were carried out with SPSS 22.0 software (IBM, Chicago, USA) and GraphPad Prism 7 software (GraphPad, Inc., La Jolla, CA, USA). All experiments were triplicated and data are indicated as mean ± standard (SD) deviation. A P-value <0.05 was considered significant.

## Results

### Bioinformatics Analysis

#### DEGs in PM of GC

We used three criteria (**Figure 1A**) to screen the TCGA and ACRG databases for genes associated with PM of GC: a. DEGs between PM patients and non-PM patients in the ACRG dataset; b. overexpressed genes associated with poor prognosis in GC patients in ACRG and TCGA datasets; c. DEGs between GC tissues and adjacent normal tissues in the TCGA data set. Through conditional screening, we found that a total of 13 genes met the criteria (**Table 1**), which were considered to be related to PM of GC. In our previous study (4), FNDC1 was found to have a higher frequency of mutations in patients with PM of GC by whole-exome sequencing (WES) of postoperative tumors and adjacent normal tissues, however the specific mechanism of action is unknown. Therefore, we aimed to further explore its specific role and mechanism.

RETRACTED

**Figure 1:** Results of Bioinformatics Analysis: **(A)** Three criteria for screening PM-related genes; **(B)** FNDC1 mRNA level of tumor *versus* normal tissue from GEPIA database; **(C)** FNDC1 mRNA level of PM *versus* non-PM tissue from TCGA database; **(D)** Relationship between FNDC1 mRNA level and OS of patients with GC based on GEO database; **(E)** Relationship between FNDC1 mRNA level and OS of patients with GC based on TCGA database.

**Table 1:** DEGs screening for PM of GC.

Gene symbol
SFRP1、 C7、 ADH1B、 BGN、 TSC22D3、 CDH11、 COL8A1、 SCUBE2、 OLFML2B、 SFRP4、 THY1、 GPX3、 FNDC1	

DEGs, differentially expressed genes; GC, gastric cancer; PM, peritoneal metastasis.

#### FNDC1 Is Up-Regulated in GC and PM Tissues and Correlates With Prognosis

We found that FNDC1 expression was significantly increased in GC tissues (T) compared with adjacent normal tissues (N) (P < 0.05). There was also a significant difference in FNDC1 expression between PM patients and non-PM patients (P = 0.011) (**Figures 1B, C**). To further compare the correlation between FNDC1 expression and prognosis, we stratified patients into groups with high FNDC1 expression and low FNDC1 expression, using KM-Plot survival analysis and log-rank test to compare survival differences. The results of both GEO dataset and TCGA dataset showed that the expression of FNDC1 in GC patients was significantly correlated with survival prognosis (P < 0.05) (**Figures 1D, E**).

#### The Expression of FNDC1 Is Correlated With Epithelial-Mesenchymal Transition

To investigate the signaling pathways regulated by FNDC1 expression, we performed GSEA analysis using TCGA and ACRG datasets (**Supplemental Figures 1A, B**), which showed that high expression of FNDC1 positively correlated with EMT in GC.

### High Expression of FNDC1 in GC Tissues

To characterize the expression of FNDC1 in the GC, IHC was performed on 74 primary GC tumor tissues and paired adjacent normal tissues. As shown in **Figure 2A**, FNDC1 expression was higher in tumor tissues than that in adjacent normal tissues. Next, we scored the results of IHC among these specimens (**Table 2**). A significant high expression of FNDC1 was observed in 66.2% (49/74) of the GC tissues, compared with the adjacent normal tissues (21.6%, 16/74), and this difference was statistically significant (P < 0.001) (**Figure 2B**).

RETRACTED

**Figure 2:** FNDC1 was overexpressed in GC tissues and associated with prognosis. **(A)** Immunohistochemistry (IHC) revealed FNDC1 expression in GC tissues (n = 74) and adjacent non-tumor tissues (n = 74). **(B)** FNDC1 staining score in GC tissues (Cancer) and adjacent normal tissues (Normal) by IHC analysis. **(C)** Disease-free survival (DFS) analysis of GC patients with high or low expression of FNDC1. **(D)** Overall survival (OS) analysis of GC patients with high or low expression of FNDC1.

**Table 2:** IHC staining score of FNDC1 in GC and adjacent normal tissues (mean ± SD).

Type	Intensity of staining	Proportion of positive cells	H-score	P value
Tumor tissues	2.86 ± 0.71	2.12 ± 0.50	6.05 ± 1.94	P < 0.001
Adjacent normal tissues	1.99 ± 0.75	2.16 ± 0.74	4.03 ± 1.66	

IHC, immunohistochemical; GC, gastric cancer; SD, standard deviation.

### Relationship Between FNDC1 Expression and Clinicopathological Characteristics

The clinicopathological characteristics with respect to FNDC1 expression from Fujian Medical University Union Hospital are summarized in **Table 3**. It was found that the expression of FNDC1 was significantly correlated with tumor size (P = 0.007), T classification (P = 0.038), N classification (P = 0.007), TNM stage (P = 0.011), and postoperative recurrence (P = 0.006). However, there were no differences in age, gender, tumor location, differentiation, vascular invasion, nerve metastasis, and Her-2 phenotype between the groups (P > 0.05).

**Table 3:** Correlation of clinicopathological features of FNDC1 in 74 patients.

Characteristics	All patients	FNDC1 expression		P value
		Low	High	
No.	74	25	49	
Age (years)				
<60	23	8	15	0.903
≥60	51	17	34
Gender				
Male	54	20	34	0.331
Female	20	5	15
Tumor location				
Upper part (cardia, fundus)	28	8	20	0.403
Middle and lower part (gastric body, pylorus)	40	16	24
Whole stomach	6	1	5
Tumor size (cm)				
<5	34	17	17	0.007
≥5	40	8	32
Differentiation				
Well-moderate	37	15	22	0.219
Poor	37	10	27
T classification				
T1+T2	32	15	17	0.038
T3+T4	42	10	32
N classification				
N0 + N1	42	19	23	0.007
N2 + N3	32	6	26
Vascular invasion				
Yes	48	15	33	0.531
No	26	10	16
Nerve invasion				
Yes	49	14	35	0.184
No	25	11	14
TNM stage				
I–II	38	18	20	0.011
III	36	7	29
Her-2				
Positive	5	2	3	0.761
Negative	69	23	46
Postoperative recurrence				
Peritoneal metastases	31	5	26	0.006
Other sites	41	18	23
No	2	2	0

RETRACTED

### Association Between FNDC1 and Prognosis

To further investigate the association between FNDC1 expression and disease-free survival (DFS) and overall survival (OS), we performed Kaplan-Meier survival analysis and log-rank test in all 74 patients. The results showed that the higher of FNDC1 expression was associated with poorer DFS (P = 0.002) and OS (P = 0.005) (**Figures 2C, D**).

Subsequently, we performed univariate and multivariate analyses for factors affecting overall survival (**Table 4**). Univariate analysis indicated that the tumor size (P < 0.001), differentiation (P = 0.04), depth of invasion (P < 0.001), lymph node metastasis (P = 0.004), TNM stage (P = 0.001), postoperative recurrence (P = 0.009), and FNDC1 expression (P = 0.005) were significantly correlated with poor OS. Furthermore, multivariate analysis showed that both depth of invasion and FNDC1 expression were independent poor prognostic marker for GC.

**Table 4:** Univariate and multivariate analysis of the association of prognosis with clinicopathologic parameters and expression of FNDC1 in GC.

Variable	Univariable analysis		Multivariable analysis	
	P value	HR (95% CI)	P value	HR (95% CI)
Age (<60 *vs.* ≥60)	0.083	1.741 (0.930–3.258)		
Sex (male *vs.* female)	0.659	0.872 (0.474–1.603)		
Tumor location	0.297	1.273 (0.809–2.002)		
Tumor size (<5 *vs.* ≥5 cm)	<0.001	2.939 (1.672–5.169)	0.558	
Differentiation (well *vs.* poor)	0.040	1.771 (1.027–3.054)	0.481	
Depth of invasion (T1–2 *vs.* T3–4)	<0.001	3.271 (1.802–5.937)	0.001	2.917 (1.596–5.333)
Lymph node metastasis (N0–1 *vs.* N2–3)	0.004	2.206 (1.286–3.786)	0.689	
Vascular invasion (Yes *vs.* No)	0.069	1.708 (0.959–3.044)		
Nerve invasion (Yes *vs.* No)	0.212	1.452 (0.809–2.607)		
TNM stage (I–II *vs.* III)	0.001	2.499 (1.451–4.305)	0.789	
Her-2 (Positive *vs.* Negative)	0.401	0.607 (0.189–1.947)		
Postoperative recurrence Peritoneal metastases Other sites No	0.009	1.960 (1.187–3.235)	0.755	
FNDC1 expression (high *vs.* low)	0.005	2.365 (1.260–4.439)	0.040	1.957 (1.032–3.713)

GC, gastric cancer.

### The mRNA Transcription and Protein Overexpression of FNDC1 *In Vitro*

qRT-PCR was used to detect the differences in mRNA transcription of FNDC1 between GC cell lines (AGS, MGC803, BGC823, HGC27) and normal gastric epithelial cell lines (GES1). The results showed that the mRNA transcription of FNDC1 was significantly increased in GC cell lines compared with GES1, with MGC803 and AGS being the most significant (P < 0.01, **Figure 3A**). Subsequently, we examined the differences in FNDC1 protein expression between GC cell lines (MGC803, AGS) and GES1 by WB. The results showed that the protein expression of FNDC1 in GC cell lines (MGC803, AGS) was significantly increased compared with GES1(P < 0.01, **Figures 3B, C**). Thus, we demonstrated that the mRNA transcription and protein expression of FNDC1 were significantly increased in GC cells compared with GES1 by *in vitro* assays.

RETRACTED

**Figure 3:** The expression of FNDC1 in GES1, AGS, HGC27, BGC823, and MGC803. The mRNA levels in different cells were measured by qRT-PCR **(A)**, and the expression of FDNC1 in different cells were detected by WB **(B, C)**. The results were presented as mean ± SD (n = 3). **p < 0.01 *vs* GES1.

### Construction of Lentivirus-Transfected GC Cells

To explore the role of FNDC1 expression in GC, we selected AGS, MGC803 and BGC823 cells as cell models. The prepared lentiviruses were used to infect AGS, MGC803, and BGC823, which were subsequently further validated by WB and qPCR (**Supplemental Figures 2**–**4**).

### FNDC1 Promotes the Proliferation, Invasion, and Migration of GC Cells

In order to understand the role of FNDC1 expression in the invasion and metastasis of GC, we transfected lentivirus into AGS and MGC803 cells for FNDC1 knockdown and followed by a series of *in vitro* assays such as CCK8, cell cycle assay, colony formation assay, invasion assay, scratch assay, and Edu staining assay.

Cell proliferation curves were measured using CCK8, and the results showed that the rate of cell proliferation was significantly increased in the AGS group compared with the GSE1 group; the rate of cell proliferation was significantly decreased in the AGS-shRNA-FNDC1 group compared with the AGS-shRNA-NC group (**Supplemental Figure 5A**). Similarly, the rate of cell proliferation was significantly increased in the MGC803 group compared with the GSE1 group; the rate of cell proliferation was significantly decreased in the MGC803-shRNA-FNDC1 group compared with the MGC803-shRNA-NC group (**Supplemental Figure 5B**).

Cell cycle was examined by flow cytometry, and the results showed that the G2 phase of cells in the AGS-shRNA-FNDC group was significantly increased compared with the AGS-shRNA-NC group (**Supplemental Figures 6A, B**). Similarly, the G2 phase of cells in the MGC803-shRNA-FNDC group was significantly increased compared with the MGC803-shRNA-NC group (**Supplemental Figures 6A, C**).

By colony formation assay, the results showed that the number of colony formation was significantly increased in the AGS group compared with the GES1 group, while AGS-shRNA-FNDC1 was significantly decreased compared with the AGS-shRNA-NC group (**Supplemental Figures 7A, B**). In addition, the number of colonies was significantly increased in the MGC803 group compared with the GES1 group, and after MGC803-shRNA-FNDC1 transfection, it was significantly decreased compared with the MGC803-shRNA-NC group (**Supplemental Figures 7A, C**).

RETRACTED

Through cell invasion assay, we found that the cell invasion ability of AGS group was significantly increased compared with GES1 group, and after AGS-shRNA-FNDC1 transfection, it was significantly attenuated compared with AGS-shRNA-NC group (**Supplemental Figures 8A, B**). Similarly, cell invasion was significantly increased in the MGC803 group compared with the GES1 group, while invasion was significantly attenuated in the transfected MGC803-shRNA-FNDC1 compared with the MGC803-shRNA-NC group (**Supplemental Figures 8A, C**).

We used scratch assay to demonstrate the effect of cell FNDC1 on cell migration, and the results showed that the cell migration ability of the AGS and MGC803 groups was significantly increased compared with the GES1 group, while the transfected AGS-shRNA-FNDC1 and MGC803-shRNA-FNDC1 groups were significantly decreased compared with the AGS-shRNA-NC and MGC803-shRNA-NC groups, respectively (**Supplemental Figures 9A–C**).

In addition, we also performed Edu staining assay, and the results showed that the cell proliferation ability of AGS and MGC803 groups was significantly increased compared with GES1 group. Moreover, the cell proliferation ability of transfected AGS-shRNA-FNDC1 and MGC803-shRNA-FNDC1 was significantly decreased compared with AGS-shRNA-NC group and MGC803-shRNA-NC group, respectively (**Supplemental Figures 10A–C**).

Through the above experiments, we demonstrated that the proliferation, migration, and proliferative activity of GC cells could be significantly inhibited by knockdown FNDC1.

### FNDC1 Regulates the Tumorigenesis of GC Cells

By knockdown FNDC1, we investigated the effect of MGC803-shRNA-FNDC1 on proliferation or inhibition of xenograft tumors in nude mice. The results are as follows: a. there was no significant difference between the body weights of mice in each group; b. there was no significant difference in the MGC803-shRNA-NC group compared with the MGC803 group; c. tumor volume and mass were significantly decreased in the MGC803-shRNA-FNDC1 group compared with the MGC803-shRNA-NC group (**Figures 4A–D**). Through *in vivo* experiments, we demonstrated that knockdown FNDC1 could significantly inhibit the proliferative activity of GC cells in xenograft tumors.

**Figure 4:** Images show tumor growth **(A)**. Influence of FNDC1 on changes of body weight **(B)** and antitumor effects **(C)** of MGC803 xenograft-bearing nude mice. Weights **(D)** of tumors resected from each group of sacrificed mice on the last day. The results were presented as mean ± SD (n = 6). **p < 0.01, *vs.* MGC803- shRNA –NC.

RETRACTED

### FNDC1 Affects the EMT Process of GC

We investigated the effects of FNDC1 on the EMT process in GC by examining the changes in the levels of EMT pathway-related proteins such as: E-cadherin, Krt12, vimentin, survivin, Snail, Slug, total β-catenin, and β-catenin in the nucleus. The results showed that E-cadherin and Krt12 protein levels were significantly increased, while vimentin, survivin, Snail, and Slug protein levels were significantly decreased in MGC803-shRNA-FNDC1 group compared with MGC803-shRNA-NC group (**Figures 5A–G**), and total β-catenin and nuclear β-catenin protein levels were also significantly decreased (**Figures 6A–C**). Moreover, we also detected the changes of EMT signaling pathway in xenograft tumors by WB and obtained the similar results (**Supplemental Figures 11A–G**). In contrast, after overexpression of FNDC1, E-cadherin and Krt12 protein levels were significantly decreased, and vimentin, survivin, Snail, and Slug protein levels were significantly increased in the BGC823-FNDC1 group compared with the BGC823-FNDC1-NC group (**Figures 7A–G**).

**Figure 5:** FNDC1 knockdown in MG803 cells weakened EMT. After transfected shRNA-FNDC1, the E-cadherin, Krt12, vimentin, survivin, Snail, and Slug expressions in MG803 cells were detected by WB assay, representative bands were shown in **(A)**. The levels of E-cadherin **(B)**, Krt12 **(C)**, vimentin **(D)**, survivin **(E)**, Snail **(F)**, and Slug **(G)** were normalized to MGC803. The results were presented as mean ± SD (n = 3). **p < 0.01, *vs.* MGC803-shRNA-NC group.

**Figure 6:** Effect of knockdown FNDC1 on the β-catenin in MGC803 cells. After transfected shRNA-FNDC1, the level of β-catenin expression was detected by WB assay, and representative bands were shown in **(A)**. The level of total β-catenin **(B)** and nucleus level of β-catenin **(C)** were normalized toMGC803. The results were presented as mean ± SD (n = 3). *p < 0.05, **p < 0.01, *vs.* MGC803-shRNA-NC group.

**Figure 7:** FNDC1 overexpression in BGC823 cells promoted EMT. After transfected, the E-cadherin, Krt12, vimentin, survivin, Snail, and Slug expressions in BGC823 cells were detected by WB assay, representative bands were shown in **(A)**. The levels of E-cadherin **(B)**, Krt12 **(C)**, vimentin **(D)**, survivin **(E)**, Snail **(F)**, and Slug **(G)** were normalized to BGC823. The results were presented as mean ± SD (n = 3). *p < 0.05, **p < 0.01, *vs.* BGC823-FNDC1-NC group.

In addition, we further added MG132 during cell culture in each experimental group and performed co-IP experiments. The results showed that β-catenin ubiquitination levels were significantly increased after transfection with shRNA-FNDC1 compared with the MGC803-shRNA-NC group (**Figures 8A, B**). To further validate the results, we overexpressed β-catenin in MGC803-shRNA-FNDC1 cells and carried out relevant rescue experiments. We found that after MGC803-shRNA-FNDC1 transfection, the number of colony formation was significantly decreased compared with the MGC803-shRNA-NC group, while overexpression of β-catenin could reverse the trend (**Supplemental Figures 12A, B**). Moreover, by scratch assay, we demonstrated that after MGC803-shRNA-FNDC1 transfection, cell migration was significantly reduced compared with the MGC803-shRNA-NC group, while overexpression of β-catenin could reverse the trend (**Supplemental Figures 13A, B**).

RETRACTED

**Figure 8:** The ubiquitin level of β-catenin in MGC803 cells. The ubiquitin level of β-catenin was measured with co-IP **(A)**. Ubiquitin level of β-catenin was normalized to MGC803 **(B)**. The results were presented as mean ± SD (n = 3). **p < 0.01, vs. MGC803-shRNA-NC group.

Through the above experiments, it is indicated that FNDC1 may be involved in the regulation of Wnt/β-catenin signaling pathway.

## Discussion

Although great advances in current treatments have improved the prognosis of GC patients, about 50% of patients still experience tumor recurrence and metastasis within 2 years after surgery and eventually die (2). PM is the most common site of metastasis in GC, but the prognosis of patients is very poor due to the limited treatment and efficacy. However, there is still a lack of effective predictors for PM. Therefore, the active search for effective molecular markers, and elucidation of the underlying molecular mechanisms deserve our continuous research, so as to provide a basis for clinical diagnosis and treatment. In recent years, the role of extracellular matrix macromolecules (ECM) in tumor invasion and metastasis has received increasing attention (18, 19). Nevertheless, as one of the main members of ECM, there are still few reports on the role and function of FNDC1 in GC.

The FNDC1 gene is closely related to many diseases. Wuensch (20) found that FNDC1 was associated with pathological changes in inflammatory bowel disease. Van (21) performed a WES study and found that FNDC1 plays an important role in the development of acute otitis media in children. FNDC1 can also participate in hypoxia-induced cardiomyocyte apoptosis by regulating G protein signaling (22). FNDC1 is also associated with vascular endothelial growth factor (VEGF)–mediated cellular events, including angiogenesis, migration, and proliferation (23). In addition, there are multiple articles reporting the role of FNDC1 in tumors. Anderegg (5) demonstrated that the expression of FNDC1 was upregulated with skin tumor progression and increased tumor thickness. Bell (6) found that FNDC1 promotes apoptosis in human sialoid cystic carcinoma by hypermethylation. Some scholars have found that the up-regulation of microRNA-1207-3p can significantly inhibit the migration and proliferation of tumors in the study of prostate cancer, further verifying that it can induce tumor cell apoptosis by regulating the downstream target gene FNDC1 (7). Recent studies have also reported a correlation between the expression of FNDC1 in GC and clinical characteristics of patients, reporting that the overexpression of FNDC1 is associated with poor prognosis of patients (8–10). In our previous study (4), molecular markers of PM were analyzed by WES and FNDC1 was found to have a higher frequency of mutations in PM patients, suggesting that FNDC1 may be associated with GC invasion and PM. Therefore, we comprehensively analyzed the effects of FNDC1 expression on GC invasion and PM using biological information analysis, gene transfection, RNA interference, proteomics, and tumor xenograft models herein.

RETRACTED

Firstly, the correlation between FNDC1, PM, and prognosis of GC was clarified by bioinformatics and clinicopathological analysis. We found that FNDC1 was highly expressed in GC and was associated with PM and poor prognosis. In addition, we also found that FNDC1 was also associated with EMT in GC cells. Next, the effect of FNDC1 expression on the invasion and metastasis ability of GC was investigated *in vivo* and *in vitro*. And it was clarified that knockdown of FNDC1 could inhibit the proliferation, invasion, and migration of GC cells. Finally, the signaling pathways involved in the regulation of FNDC1 were explored. Through a series of proteomics experiments, it was elucidated that FNDC1 promotes EMT through the Wnt/β-catenin signaling pathway.

Shedding of tumor cells from the primary site is the first step of tumor invasion and metastasis, which is associated with reduced cell adhesion, and EMT is an important cause of reduced tumor cell adhesion (24, 25). Triggering of EMT mechanisms is often accompanied by changes in cell morphology as well as molecular markers in tumor cells. EMT is also able to cause some ECM and basement membrane degradation, which effectively disrupts the formation of histological barriers that block tumor cell invasion. Thus, the tumor cells are detached from the primary site in an intact structure and invade and metastasize to surrounding or distant normal tissues. The process of EMT mechanism in tumor cells is highly correlated with numerous signal transduction pathways as well as multiple regulators. Among them, Wnt/β-catenin signaling pathway plays an important role in EMT of GC cells (26). Wnt/β-catenin signaling pathway is one of the most important signaling pathways leading to the development and progression of GC. For the digestive system, Wnt/β-catenin signaling pathway not only regulates cell proliferation and differentiation, but also regulates the biological activity of stem cells. The Wnt/β-catenin pathway is conducted as follows: ligand proteins bind to frizzled (FDZ) and LRP5/6 proteins to form trimers, causing diminished stability of complexes composed of Axin, GSK-3β, and APC in the cytoplasm, which leads to reduced ubiquitination of β-catenin. In this way, β-catenin protein continuously accumulates and translocates into the nucleus to further activate downstream target genes (27). Central to the activation of the Wnt/β-catenin signaling pathway is the accumulation of β-catenin in the cytoplasm followed by nuclear transfer, while changes in any component of the pathway can lead to abnormal signal transduction. In our study, the expression of FNDC1 was found to have a certain impact on several key proteins for EMT development and Wnt/β-catenin signaling pathway.

RETRACTED

Mechanistically, FNDC1 is not a typical intracellular expression protein, which is mainly expressed in the nucleus and extracellular matrix, in other words, FNDC1 is also a secreted protein. We combed all relevant literature on FNDC1 and found that there is currently a paucity of literature on FNDC1. Existing studies have mainly analyzed FNDC1 as a protein of the extracellular matrix and rarely investigated its role within the nucleus. We obtained important information from various literatures: FNDC1 can bind to the Gβγ subunit in G proteins (22, 23), which can potentially regulate the sustained activation and shutdown of the Wnt/β-catenin signaling pathway (28). As shown in **Supplemental Figure 14** (29), when Wnt family ligands bind to FDZ and LRP5/6 complexes, they recruit intracellular Dvl and Axin. Recruitment of Dvl and Axin prevents Axin from forming the Axin-GSK3β complex, which continuously mediates ubiquitination of β-catenin in the unactivated state of the Wnt/β-catenin signaling pathway, resulting in its degradation by proteases. Ultimately, this action hinders β-catenin as a core transcription factor-mediated downstream gene activation. Axin is alternatively recruited to form a complex with LRP5/6 and Gβγ, at which point Axin is labeled by ubiquitination and degraded. Subsequently Gβγ can then bind to Dvl and induce Dvl ubiquitination, leading to its degradation and ultimately the blockage and inactivation of the Wnt/β-catenin signaling pathway. Gβγ plays an important role in the normal dynamic process of receptor activation and inactivation. Specifically, recruitment of the initiating Dvl and Axin leads to activation of Wnt/β-catenin, followed by Gβγ mediated degradation of Dvl, resulting in reclosure of the Wnt/β-catenin signaling pathway. Therefore, we speculated that FNDC1 could bind to Gβγ on the cell membrane and form a complex with LRP5/6 and Gβγ, hindering Gβγ-mediated inactivation of Wnt/β-catenin signaling pathway by inhibiting the binding of Gβγ to Dvl. In our subsequent experiments, the specific regulatory mechanism of FNDC1 in the Wnt/β-catenin signaling pathway will be intensively studied.

RETRACTED

## Conclusion

In summary, the results of our study suggest that FNDC1 promotes the invasiveness of GC *via* Wnt/β-catenin signaling pathway and correlates with PM and prognosis. FNDC1 was highly expressed in GC tissues and cell lines, while its high expression was also significantly associated with poor DFS and OS. Both univariate and multivariate analyses suggested that the expression of FNDC1 was an independent factor for GC. Knockdown of FNDC1 significantly inhibited the proliferation, migration, and activity of GC cells. FNDC1 may promote EMT in GC cells through the regulation of Wnt/β-catenin signaling pathway, and it is of great potential significance to further explore its specific regulatory mechanism, which we expect to explore subsequently. FNDC1 has the potential to be used as a predictor of PM and can also be studied in depth as a therapeutic target for GC, which has potential clinical utility and is worthy of further validation.

## Data Availability Statement

The raw data supporting the conclusions of this article will be made available by the authors, without undue reservation.

## Ethics Statement

The studies involving human participants were reviewed and approved by the Fujian Medical University Union Hospital Ethics Committee. The patients/participants provided their written informed consent to participate in this study. The animal study was reviewed and approved by the Institutional Review Board (IRB number: 2020KJT022) of Fujian Medical University Union Hospital. Written informed consent was obtained from the individual(s) for the publication of any potentially identifiable images or data included in this article.

## Author Contributions

All named authors meet the International Committee of Medical Journal Editors (ICMJE) criteria for authorship for this article, take responsibility for the integrity of the work as a whole, and have given their approval for this version to be published. TJ, XL, and QC conceptualized and supervised the study, contributed to the methodology, software, writing and preparing of the original draft, and reviewing, editing, and approving the manuscript. WG, SL, HC, BD, and QL contributed to the data curation, visualization, investigation and validation, and reviewing and approving the manuscript. All authors contributed to the article and approved the submitted version.

RETRACTED

## Funding

The study was funded by the Joint Funds for the Innovation of Science and Technology Fujian Province (2018Y9031 and 2018Y9032).

## Conflict of Interest

The authors declare that the research was conducted in the absence of any commercial or financial relationships that could be construed as a potential conflict of interest.

## Supplementary Material

Supplementary Figure 1 Analysis of the TCGA **(A)** and ACRG **(B)** datasets using GSEA showed a positive correlation between the expression of FNDC1 and EMT.

Supplementary Figure 2 Knockdown of FNDC1expression in GC cells. WB analysis showed the efficiency of FNDC1 knockdown in AGS **(A)** and MGC803 **(B)** cells. The levels of FNDC1 were indicated as folds of control **(C, D)**. The results were presented as mean ± SD (n = 3). **p < 0.01, *vs.* control group.

Supplementary Figure 3 Effect of the mRNA expressions of FNDC1 in BGC823 cell. The mRNA levels of FNDC1 was detected by qRT-PCR. The mRNA levels of FNDC1 were normalized to BGC823. The results were presented as mean ± SD (n = 3). **p < 0.01, *vs.* BGC823-FNDC1-NC group.

Supplementary Figure 4 Effect of the mRNA expressions of β-catenin in MGC803 cell. The mRNA levels of β-catenin were detected by qRT-PCR. The mRNA levels of β-catenin were normalized to MGC803. The results were presented as mean ± SD (n = 3). **p < 0.01 *vs.* MGC803-shRNA-FNDC1+β-catenin NC.

Supplementary Figure 5 FNDC1 shRNA weakened cell viability in AGS **(A)** or MGC803 **(B)**. Cells viability were measured with CCK-8 assay after 24, 48, and 72 h incubation. The results were presented as mean ± SD (n = 5). **p < 0.01 *vs.* GES1 group. ##p < 0.01 *vs.* AGS-shRNA-NC group or MGC803-shRNA-NC group.

Supplementary Figure 6 FNDC1 shRNA inhibited growth of GC cells by inducing G2-M arrest. Flow cytometry with propidium iodide staining for AGS **(A, B)**, MGC803 **(A, C)**, or GES1 after 48 h. **p < 0.01 vs. GES1 group. ##p < 0.01 vs. AGS shRNA-NC group or MGC803-shRNA-NC group.

Supplementary Figure 7 Knockdown of FNDC1 inhibit colony formation of GC. Colony formation assay showed that knockdown of FNDC1 inhibited cell invasion of AGS and MGC803 **(A)**. Graphical representation of the number of invasive AGS **(B)** and MGC803 **(C)** cells per microscopic field. Data were shown as the mean ± SD from three independent experiments. **p < 0.01 **vs.** GES1 group. ##p < 0.01 **vs.** AGS-shRNA-NC group or MGC803-shRNA-NC group.

RETRACTED

Supplementary Figure 8 Knockdown of FNDC1 inhibited the invasion of gastric cell in vitro. Transwell invasion assay showed that knockdown of FNDC1 inhibited cell invasion of AGS and MGC803 **(A)**. Graphical representation of the number of invasive AGS **(B)** and MGC803 **(C)** cells per microscopic field. Data were shown as the mean ± SD from three independent experiments. **p < 0.01 *vs.* GES1 group. ##p < 0.01 *vs.* AGS-shRNA-NC group or MGC803-shRNA-NC group.

Supplementary Figure 9 Knockdown of FNDC1inhibit wound healing in GC cells. AGS and MGC803 cells were transfected with shRNA-NC or shRNA-FNDC1. Movement of cells into wound was shown for AGS and MGC803 cells at 0 and 72 h **(A)**. The lines indicated the boundary lines of scratch. Cell migration was assessed by recover of the scratch. Graphical representation of the number of invasive AGS **(B)** and MGC803 **(C)** cells per microscopic field. Data were shown as the mean ± SD from three independent experiments. **p < 0.01 *vs.* GES1 group. ##p < 0.01 *vs.* AGS-shRNA-NC group or MGC803-shRNA-NC group.

Supplementary Figure 10 Edu assay of gastric cells. The proliferating nuclei were stained red with Edu, the nuclei of all cells were stained blue with Hoechst for 2 h. Three random pictures per group from confocal microscopy were used to count the cell numbers of Edu positive cells and Hoechst positive cells **(A)**. Data were shown as the mean ± SD from three independent experiments **(B, C)**. **p < 0.01 vs. GES1 group. ##p < 0.01 vs. AGS-shRNA-NC group or MGC803-shRNA-NC group.

Supplementary Figure 11 FNDC1 knockdown in MG803 cells weakened EMT in xenograft tumors. After transfected shRNA-FNDC1, the E-cadherin, Krt12, vimentin, survivin, Snail, and Slug expressions in MG803cells were detected by western blot assay, representative bands were shown in **(A)**. The levels of E-cadherin **(B)**, Krt12 **(C)**, vimentin **(D)**, survivin **(E)**, Snail **(F)**, and Slug **(G)** were normalized to MGC803. The results were presented as mean ± SD (n = 3). **p < 0.01, *vs.* MGC803-shRNA-NC group.

Supplementary Figure 12 Overexpression of β-catenin enhancement colony formation of GC. Transwell invasion assay showed that overexpression of β-catenin enhancement cell invasion of MGC803 **(A)**. Graphical representation of the number of invasive MGC803 **(B)** cells per microscopic field. Data were shown as the mean ± SD from three independent experiments. **p < 0.01 *vs.* MGC803-shRNA-NC group, #p < 0.05 *vs.* MGC803-shRNA-FNDC1+β-catenin NC.

RETRACTED

Supplementary Figure 13 Overexpression of β-catenin enhancement wound healing in GC. Movement of cells into wound was shown for MGC803 cells at 0 and 72 h **(A)**. The lines indicated the boundary lines of scratch. Cell migration was assessed by recover of the scratch. Graphical representation of the number of invasive MGC803 **(B)** cells per microscopic field. Data were shown as the mean ± SD from three independent experiments. **p < 0.01 *vs.* MGC803-shRNA-NC group, ##p < 0.01 *vs.* MGC803-shRNA-FNDC1+β-catenin NC.

Supplementary Figure 14 Gβγ is involved in regulating the activation and closure of the Wnt/β-catenin signaling pathway.
